# An efficient method for FITC labelling of proteins using tandem affinity purification

**DOI:** 10.1042/BSR20181764

**Published:** 2018-12-11

**Authors:** Lalith K. Chaganti, Navneet Venkatakrishnan, Kakoli Bose

**Affiliations:** 1 Advanced Centre for Treatment, Research and Education in Cancer (ACTREC), Tata Memorial Centre, Kharghar, Navi Mumbai 410210, India; 2 Homi Bhabha National Institute, Training School Complex, Anushaktinagar, Mumbai 400094, India

**Keywords:** dialysis, FITC labelling, protein stability, Tandem affinity purification

## Abstract

Fluorescence-based assays are extremely diverse, sensitive and robust experimental methods for investigating the conformational changes, enzyme kinetics, dynamics and molecular interactions. A prerequisite for most of these experimental approaches is to label the protein of interest with one or more extrinsic fluorophores with desired photophysical properties. Fluorescein isothiocyanate (FITC), due to its high quantum efficiency and conjugate stability, is most widely used fluorescence labelling reagent for such experimental approaches. However, the bottlenecks in this labelling reaction is requirement of high protein concentration, maintenance of protein stability during the labelling process as well as high background fluorescence due to ineffective removal of unreacted FITC, prior to fluorescence studies. Therefore, to overcome these inadequacies or limitations, we have modified the existing protocol by introducing tandem affinity purification tags at the N- and C-terminus of target protein. Using this modified method, we have efficiently labelled target protein with significant decrease in precipitation, degradation and background fluorescence of unreacted FITC. This facile and rapid technique may also be used as a basis for labelling procedures with other fluorophores and hence has a broad application in spectroscopic studies.

## Protocol background

Proteins are often chemically modified by covalent conjugation to investigate the conformational dynamics, molecular interactions and enzyme kinetics in order to gain insight into their biological functions [1,2]. Many single-molecule *in vitro* biochemical and cell-based experimental techniques primarily exploit fluorescence as a tool to investigate these biological functions. An essential requirement to these experimental approaches is to label one or more fluorophores on the desired protein with the required photophysical properties. Many labelling methods have been developed and utilized, including chemical modification of amino acid side chains through covalent or non-covalent binding, incorporation of unnatural amino acids and affinity labelling.

Fluorescein isothiocyanate (FITC) is the most widely used fluorescence labelling reagent for such experimental approaches due to its high quantum efficiency and conjugate stability [3–5]. FITC reacts with a primary amine on the protein to form a covalent amide bond. FITC-labelled protein substrates/peptides, antibodies, peptide hormones are used as specific probes in enzyme kinetics, immunocytochemistry as well as flow cytometry and identification of receptors on target cells, respectively. However, the success of fluorescence labelling is contingent upon several stringent factors including requirement of pure protein and high protein concentration. Moreover, slight protein aggregation or precipitation that is observed in majority of the cases at higher protein concentrations might lead to failure of the experiment. In addition, high background fluorescence due to the ineffective removal of unreacted FITC, prior to fluorescence studies, is also a major obstacle in this process [3–5].

Size-exclusion chromatography is commonly used for the removal of unreacted FITC molecules; however, this process is accompanied with the loss of proteins and undesired dilution of the sample, especially when a small quantity of proteins is labelled. Therefore, a specific and efficient FITC labelling technique is essential to overcome these inadequacies. Hence, we have modified the existing protocol by introducing tandem affinity purification (TAP) tags at the N- and C-termini of the target protein. The TAP method provides a high level of purification of the desired proteins without any contamination. The commercially available pMALc5E vector was modified in our lab for TAP, and it consists of two different affinity tags at the N- and C-terminus of the desired protein (Figure 1A,B). Maltose-binding protein (MBP) is present at the N-terminus that allows first-step purification of the fusion protein using amylose resin. Downstream to the MBP, tobacco etch virus (TEV) protease cleavage-site (ENLYFQ/G) was introduced to facilitate the separation of MBP from the target protein. The TEV protease that is often used for easy tag removal is a highly site-specific cysteine protease found in Tobacco Etch Virus [6]. Due to its stringent sequence specificity and activity over a broad temperature range (4–37°C), TEV is considered a very useful reagent for cleaving fusion proteins and better than other commercially available proteases such as factor Xa, thrombin and enterokinase. Moreover, TEV is relatively easy to overproduce and purify in large quantities. The protein of interest will also have a C-terminal His_6_ tag for efficient second-step purification using immobilized metal affinity chromatography resin.

**Figure 1:** Representation of Tandem affinity tag vector (**A**) Commercially available pMAL c5E vector with MBP tag and enterokinase cleavage-site (highlighted in red). (**B**) Modified pMAL c5E with MBP tag, TEV cleavage-site (highlighted in red) and His tag were introduced using site-directed mutagenesis kit. MBP represents maltose-binding protein, TEV is a Tobacco Etch Virus, MCS is the multiple cloning site. Blue arrow indicates the preferred scissile bonds of enterokinase and TEV protease. X is any amino acid.

Having an MBP-tag has several advantages such as it enhances the expression level, improves solubility and proper folding of its fusion partner with typical yields of 10 to 30 mg fusion protein per litre culture [7–9]. Additionally, the MBP fusion system also includes ease of purification and mild elution conditions, which are highly efficient and compatible with most downstream applications. The use of the second-step purification by His_6_ at the C-terminal region removes remaining contaminants from the first purification step.

With the help of this modified method, we have efficiently labelled target protein with a significant decrease in precipitation and degradation (Figure 2). Furthermore, second-step purification of labelled protein by His_6_ tag substantially removed the residual FITC and thus decreased the background fluorescence of unreacted FITC. Therefore, this optimized technique may also be used as a basis for labelling procedures with other fluorophores for high-throughput spectroscopic analysis of biological functions of macromolecules.

**Figure 2:** Schematic representation of FITC labelling of target protein using tandem affinity tag method

## Method details

### Step 1: Cloning

For TAP tag, modify pMALc5E vector by introducing TEV recognition cleavage-site between N-terminus of MBP and MCS. Insert His_6_ tag at the C-terminal region of the vector (Figure 1B).

#### Materials required

*Escherichia coli* DH5α (New England Biolabs (NEB), Ipswich, MA, U.S.A.), pMAL c5E (NEB), Plasmid miniprep kit (Sigma chemicals, St. Louis, MO, U.S.A.), Quick-change site-directed mutagenesis kit (Stratagene, Cedar Creek, TX, U.S.A.), Ampicillin sodium salt (Sigma), Primers (Sigma), DpnI enzyme (Fermentas, Waltham, Massachusetts, United States), IPTG (Sigma), Luria-Bertani (LB) broth (Himedia, Mumbai, India).

#### Method

- Design primers (Table 1) for introducing TEV recognition cleavage-site using ‘*primer-X’* software and ‘*oligoanalyser’* tools.
- Perform insertion mutagenesis using the quick change site-directed mutagenesis kit.
- Incubate the amplified PCR products with DpnI enzyme at 37°C for 3 h to degrade the parental template.
  Note: DpnI is an endonuclease, which specifically degrades the methylated parental DNA strands.
- Transform the digested PCR products into *E. coli* DH5α cells. Isolate the plasmids from the transformed colonies using plasmid miniprep kit.
- Confirm the insertion of TEV recognition site using automated DNA sequencing. This modified vector is now represented as pMALc5E-TEV vector.
- Similarly, introduce His_6_ tag downstream to the MCS of pMALc5E-TEV vector using the forward and reverse primers as mentioned in Table 1. Confirm the insertion of His_6_ using DNA sequencing.
  Note: This modified pMAL vector is now represented as pMALc5E-TEV-His or TAP vector.
- Sub-clone the gene of interest into the MCS of TAP vector. Confirm the clone by restriction digestion and DNA sequencing.
  Note: In our study, we have sub-cloned phosphoprotein enriched in astrocytes (Pea15) gene. Pea15 is a 15 kDa ubiquitously expressed antiapoptotic cytosolic protein with an N-terminal death effector domain (DED) and an irregularly structured C-terminal tail. Pea15, by virtue of its DED, binds to other DED-containing proteins and inhibits Fas/TNFR1-induced extrinsic apoptosis [10]. This protein was labelled to be used as a substrate in an enzyme kinetics study.

**Table 1:** Primer sequences for inserting TEV and His tag

Primer	5′ to 3′ sequence
His_6_ forward primer	CCCTGCAGGT**CACCACCACCACCA** CCACAATTAAATAA
His_6_ reverse primer	TTATTTAATT**GTGGTGGTGGTGGTGGTG**ACCTGCAGGG
TEV forward primer	GACAAGGTACCG**GAGAATCTTTATTTTCAGGGC**CATATG GCCG
TEV reverse primer	CGGCCATATG**GCCCTGAAAATAAAGATTCTC**CGGTACCTTGTC

Nucleotide sequences of TEV cleavage-site and His tag are highlighted in bold.

### Step 2: Protein expression and purification:

In our study, all recombinant proteins were expressed in bacterial protein expression system because they are easy to culture, grow fast, homogeneous, and give high yields of recombinant protein.

Note:

- *E. coli* Rosetta2 DE3 host strain should be used for expression of eukaryotic proteins that contain codons rarely used in *E. coli.*
- If the desired protein is insoluble, co-express the gene with commercially available GroEL/GroES chaperonin plasmids or use purification from inclusion bodies [11–13].

#### Materials required:

*E. coli* BL21(DE3) competent cells (NEB), Amylose beads (MERK, Darmstadt, Germany), Maltose (Sigma), LB broth, Lysis buffer (20 mM NaH_2_PO_4_/Na_2_HPO_4_ pH 8, 100 mM NaCl, 5 mM BME and 0.1% Triton-X 100), Buffer A (20 mM NaH_2_PO_4_/Na_2_HPO_4_ pH 8, 100 mM NaCl, and 2 mM β-mercaptoethanol or BME), Isopropyl β-D-1-thiogalactopyranoside (IPTG) (Sigma), Econo column (Bio rad, Hercules, California, U.S.A.)

#### Method:

- Transform 100 ng of pMALc5E-TEV-His construct into *E. coli* BL21(DE3) competent cells.
- Pick a single colony from the transformed LB agar plate and inoculate into 10 ml of LB broth containing antibiotics (100 μg/ml ampicillin) according to the host cells and plasmid construct.
- Incubate the culture overnight at 37°C for 16–18 h under continuous shaking at 200 rpm.
- After optical density (OD) reaches 0.6, inoculate 10 ml of the culture into 1 L (∼1:100 ratio of culture to media) of LB broth containing the required antibiotics and incubate at 37°C for approximately 3 h until OD reaches 0.6.
  Note: Time for OD_0.6_ values may vary for other culture mediums and strains.
- After the required incubation period, incubate the culture additionally for approximately 1 h at 18°C.
  Note: This step will increase the expression of recombinant protein.
- Induce protein expression by adding IPTG to a final concentration of 0.5 mM.
  Note: IPTG concentration may vary (between 0.1 and 1 mM) for other proteins.
- Post IPTG induction; incubate the culture at 18°C for 16 to 18 h under continuous shaking conditions.
- After 18 h, harvest the cultures at 10000 rpm for 40 min at 4°C. Discard the supernatant and proceed for protein purification or preserve the pellets at −80°C for future use.
  Note: Check protein expression before proceeding for purification.
- Initially, purify recombinant protein by MBP-tagged column purification method as described below.
- Lyse the cells by re-suspending pellet in 10 ml of lysis buffer followed by sonication and centrifugation at 10000 rpm for 20 min at 4°C. Discard the pellet and transfer supernatant (lysate) into fresh tube.
- Take 5 ml of amylose beads in 1 × 10 cm econo column and equilibrate the column with 5 column volumes (CV) of *Buffer A*.
  Note: Econo columns are high quality commercially available chromatography columns.
- After equilibration, add lysate and keep it for column binding at 4°C for 1 h under gentle shaking condition.
- After 1 h, collect the flow through and wash amylose beads with 3 CV of Buffer A.
- Elute bound proteins using elution buffer containing *Buffer A* + 10 mM maltose.
- Estimate the purity of the protein samples by loading them on 12% SDS-PAGE gel.
- Use >95% pure MBP fused target protein for FITC labelling.

### Step 3: Protein labelling:

Since the isothiocyanate group reacts with amino terminus and free primary amines in proteins, therefore, dialyse the target protein in alkaline buffer of pH 9 to generate free amino groups. This is a crucial step and should be performed prior to labelling.

Note: Do not use buffers containing free amino groups, such as tris, glycine, sodium azide etc., as they might interfere with labelling.

#### Materials required:

FITC (Sigma), Dimethyl sulphoxide (DMSO) (Sigma), 10 kDa cutoff dialysis membrane (Thermo fisher scientific, Waltham, Massachusetts, U.S.A.), 50 mM Na_2_CO_3_/NaHCO_3_ buffer pH 9 (carbonate buffer) and 100 mM NH_4_Cl.

#### Method:

- Collect all protein elutes and pool them into a single tube and concentrate the protein to 2–4 mg/ml.
- Prepare 500 ml of fresh carbonate buffer (do not store for more than 3 days).
- Dialyse 5 ml of concentrated protein solution against 500 ml of carbonate buffer for 16 h at 4°C with slow stirring.
- After 16 h, collect the protein sample from the dialysis bag and transfer it to a 15 ml centrifuge tube. Centrifuge it at 4000 rpm for 10 min at 4°C to check for precipitation; later transfer the supernatant into a fresh tube.
- Check absorbance of the samples before and after dialysis.
  Note: Check for protein degradation by loading the sample on SDS-PAGE (Figure 3B).
- Dissolve FITC in anhydrous DMSO at 1 mg/ml concentration. This should be prepared fresh for each labelling reaction.
- Add 5 μl of the dye to the dialysed protein (5 ml) every 30 min to get a final concentration of 100 ng FITC/1 μg protein. Perform this step by gently rocking the protein solution at 4°C for 12 h.
  *Precautionary measures:*
  - FITC solution should be kept in dark or wrapped in aluminium foil. Make fresh FITC solution each time and do not re-use.
  - Final DMSO concentration in the solution should be less than 10%.
  - Adding FITC slowly to protein reduces precipitation of protein.
  - All the labelling procedures should be performed under dark condition.
- Incubate this reaction setup in dark at 4°C for 12 h.
- Post 12-h incubation; centrifuge the labelled protein at 10000 rpm for 10 min at 4°C.
- Transfer the supernatant to a fresh tube and cover it with an aluminium foil.
- Perform extensive dialysis against 1 L of Buffer A for 15 h at 4°C in dark and constant gentle magnetic stirring conditions. Change the dialysis buffer every 4 h.

**Figure 3:** Protein purification using tandem affinity tags (**A**) Purification of MBP-tagged Pea15 using amylose resin. About 10 mM maltose elutes are highlighted in the rectangular box. (**B**) MBP-tagged Pea15 fractions after dialysing against 50 mM carbonate buffer (Na_2_CO_3_/NaHCO_3_) pH 9. (**C**) Purification of FITC labelled Pea15 using Ni-IDA affinity chromatography. Pea15 elutes from fractions containing 250 mM imidazole are highlighted in the rectangular box. All proteins were analysed on 15% SDS-PAGE followed by coomassie staining. (**D**) Dialysed FITC labelled Pea15 elute.

Note: This step is performed to remove unreacted FITC.

- Transfer the dialysed labelled protein into a fresh tube and centrifuge it at 10000 rpm for 10 min at 4°C to remove precipitate if any.

### Step 4: Ni-IDA metal affinity column purification:

This second step of purification is performed to remove the MBP tag, residual FITC as well as to increase the purity of the labelled protein.

#### Materials required:

TEV protease (1 mg/ml), Ni-IDA resin (MERK), Imidazole (sigma)

Note: This purification should be carried out under dark condition.

- To the labelled protein, add TEV protease (1 µg of TEV for 10 µg of protein) and incubate the reaction mixture at 18°C for 12 h. Check for the tag cleavage by analysing the sample on 15% SDS-PAGE.
- After complete cleavage, centrifuge the protein sample at 14000 rpm for 30 min at 4°C. Transfer the supernatant to a fresh falcon tube wrapped in an aluminium foil.
- Separate the MBP tag from the target protein by passing it through the Ni-IDA affinity resin.
- Take 5 ml of Ni-IDA beads in 1 × 10 cm econo column and cover it with an aluminium foil. Do not expose the resin or protein to light.
- Equilibrate the column in 5 CV of Buffer A.
- After equilibration, add labelled protein and keep it for binding at 4°C for 1 h under gentle shaking.
- Collect flow through and wash the column with 10 CV of Buffer A.
- Elute bound protein using elution buffer containing Buffer A + imidazole gradient (50–250 mM).
  Note: Collect the imidazole protein elutes in eppendrofs wrapped in aluminium foil. At this stage, protein elutes appear orange in colour (Figure 3D) suggesting that FITC is bound to the protein.
- Pool pure fractions and dialyse against Buffer A in dark condition at 4°C for 12 h to remove imidazole.
- After 12 h, check the labelling efficiency using the following formula:
  (1) $$\text{Protein concentration}=\frac{\text{A}280-(\text{A}495\times \text{CF})}{\varepsilon \text{ of protein}}\times \text{dilution factor}$$
  Where *ε* is molar extinction coefficient, *A*_280_ is absorbance of protein at 280 nm, *A*_495_ is absorbance at 495 nm, CF is correction factor = *A*_280_/*A*_max_
  (2) $$\text{Moles of FITC per mole of protein}(\text{F}/\text{P})=\frac{\text{Amax of labelled protein}}{\varepsilon \text{ of FITC}\times \text{Protein concetration}(\text{M})}\times \text{dilution factor}$$
  *ε* of FITC is 70,000 M^−1^ cm^−1^,
- Preserve the purified labelled proteins at −20°C for future use.
  Note: Purified protein can be stored for 2 to 3 months depending on the protein stability.

### Step 5: Method validation

#### Materials required:

Trypsin singles (Sigma), FITC labelled protein, Cytation-5 multimode plate reader (BioTek instruments, Winooski, VT, U.S.A.), Bovine serum albumin (BSA) (Sigma)

#### Method:

The described method has been used to effectively label an MBP-tagged Pea15 for quantitative enzyme kinetics study. Using our improved procedure, we have obtained approximately 3mg/ml of ∼95% pure FITC-labelled MBP tagged Pea15 with a significant decrease in degradation, precipitation (Figure 3A,B). Furthermore, MBP tag was successfully separated using the TEV protease followed by nickel affinity chromatography (Figure 3C,D). This second step of purification yielded approximately 97% pure labelled Pea15. Moreover, FITC labelling efficiency was found to be >90%. Hence, our results demonstrate that a TAP tag represents an attractive fusion construct for *in vitro* labelling of high levels of soluble recombinant proteins. Furthermore, labelled Pea15 was evaluated by monitoring the proteolytic cleavage of FITC-Pea15 using trypsin, which is a pancreatic serine protease. Trypsin specifically cleaves substrates at the carboxyl side of lysine and arginine amino acids.

##### Trypsin protease assay method:

FITC-Pea15 substrate cleavage was determined by incubating 50 nM of enzyme with 5 µM of labelled protein at 37°C for 30 min in Buffer A. Proteolytic cleavage was assessed by monitoring increase in fluorescence intensity of unquenched FITC in Cytation 5 multi-well plate reader at 485 nm excitation and 535 nm emission wavelengths [14]. In this protease assay, BSA was used as a negative control.

##### Result:

FITC labelled protein cleavage with a concomitant increase in fluorescence of unquenched FITC was observed in a time-dependent manner without any background FITC fluorescence (Figure 4). No increase in fluorescence was observed in the negative controls. Hence, our improved protocol proved to be a substantially better method than the conventional protocol.

**Figure 4:** Protease assay with trypsin using FITC Pea15 as a substrate Increase in fluorescence of unquenched FITC was recorded at 485 nm excitation and 535 nm emission wavelengths. BSA has been used as negative control.

## Discussion

In the present study, we have modified the conventional FITC labelling protocol by introducing the TAP tags at the N- and C- termini of the target protein. We have also modified the commercially available pMALc5E plasmid vector to enhance protein homogeneity, concentration, and labelling efficiency. We accomplished this by introducing MBP at the N-terminus and His_6_ tag at the C-terminus regions of the target protein. In addition, we replaced the enterokinase cleavage-site (DDDDK/X) with a more specific TEV cleavage-site (ENLFYQ/G) in vector for tag separation.

Previously, our effort to label the target protein with FITC using conventional protocol resulted in excessive protein degradation, precipitation, and high residual FITC background during the dialysis and labelling processes [3–5]. This consequently led to an insufficient yield of labelled protein with lower final concentration (∼0.5 mg/ml) that limited its use for qualitative protease assays. Moreover, to remove the 45 kDa MBP tag and the residual FITC from the labelled protein, we initially attempted cleavage with TEV and subjected it to gel filtration chromatography. However, during this purification process, the overall yield of labelled protein decreased significantly and hence to circumvent these problems, we have modified the conventional labelling protocol by cloning target gene in TAP tag vector. These modifications enabled the purification of 2 mg/ml of FITC labelled protein at over 97% homogeneity from a starting culture volume of 250 ml with a significant decrease in protein precipitation and degradation.

Hence, this TAP tag fusion system offers an attractive method for purification and labelling of several difficult eukaryotic and prokaryotic proteins. To avoid interference of large MBP tag (45 kDa) on the target protein functions if any, several other small-sized tags like glutathione-S-transferase, thioredoxin (GST), streptavidin etc. can be used for TAP tag purification. Appropriate vectors coding these tags are commercially available. In addition, our improved labelling protocol can also be employed for purification and labelling of proteins from inclusion bodies even in the presence of MBP tag. These inclusion bodies can be initially purified under denaturing conditions using the His_6_ tag and subsequently refolded and labelled [15]. During this process, the N-terminal MBP will aid in stabilizing the target protein and eventually increase the yield of the protein. Further, refolded protein can be labelled and purified to homogeneity using the second-step purification.

In addition to FITC conjugation, this improved procedure can also be used for labelling other amine (succinimidyl esters), thiol reactive (IAEDANS, monobromobimane, maleimide etc.), and biotin conjugates for studying enzyme kinetics, protein–protein interactions, conformational changes, and dynamics. Therefore, our improved labelling procedure is well suited for high throughput spectrosopic analysis for a wide variety of studies.

## Abbreviations

FITC: fluorescein isothiocyanate
MBP: maltose-binding protein
TAP: tandem affinity purification
TEV: tobacco etch virus
